# Correlation of CT Perfusion Parameters and Vascular Endothelial Growth Factor (VEGF) and Basic Fibroblast Growth Factor (BFGF) in Patients with Primary Liver Cancer

**DOI:** 10.1155/2022/4548922

**Published:** 2022-05-24

**Authors:** Xiao-min Li, Wei-bin Chen, Jing Zhang, Li-fang Ma, Qiang Li, Chao Feng, Xian-hua Yuan, Li-qing Kang

**Affiliations:** ^1^Department of Radiology, The First Affiliated Hospital of Xingtai Medical College, Xingtai, Hebei Province, China; ^2^Graduate School, Tianjin Medical University, Tianjin 300070, China; ^3^North China University of Science and Technology, Tangshan, Hebei 063000, China; ^4^Department of Hematology, The First Affiliated Hospital of Xingtai Medical College, Xingtai, Hebei Province, China; ^5^Department of Medical Imaging, Cangzhou Central Hospital, Cangzhou Teaching Hospital ofTianjin Medical University, Cangzhou, Hebei 061001, China

## Abstract

**Objective:**

To investigate the correlation of CT perfusion-related parameters with serum vascular endothelial growth factor (VEGF) and basic fibroblast growth factor (BFGF) in patients with primary liver cancer.

**Methods:**

A total of 100 patients with primary liver cancer who were treated in our hospital from June 2019 to June 2021 were selected as the observation group, and 90 patients with benign liver lesions during the same period were selected as the control group. The CT perfusion-related parameters (perfusion volume and perfusion index) and serum VEGF and BFGF levels were compared between the two groups. Pearson correlation was used to analyze the correlation between CT perfusion-related parameters and serum VEGF and BFGF levels.

**Results:**

Compared to the control group, significantly higher HAP and lower HPP and TLP were observed in the observation group. The perfusion volume indexes of patients with different stages of liver cancer in the observation group were statistically different (*P* < 0.05). Compared to the control group, the observation group witnessed significantly higher HAPI and lower HPPI. There were statistically significant differences in the perfusion index of patients with different stages of primary liver cancer in the observation group (*P* < 0.05). The serum VEGF and BFGF levels in the observation group were significantly higher than those in the control group, and the serum VEGF and BFGF levels in patients with different stages of primary liver cancer in the observation group were statistically different (*P* < 0.05). Pearson correlation analysis showed that HAP and HAPI were positively correlated with VEGF and BFGF (*r* = 0.986, *P* ≤ 0.001; *r* = 0.983, *P* ≤ 0.001), and HPP, TLP, and HPPI were negatively correlated with VEGF and BFGF (*r* = −0.992, *P* ≤ 0.001; *r* = -0.993, *P* ≤ 0.001; *r* = −0.995, *P* ≤ 0.001).

**Conclusion:**

CT perfusion-related parameters and serum VEGF and BFGF levels in patients with primary liver cancer are abnormally expressed, and there is a strong correlation between the two, which might aid clinical diagnosis and treatment.

## 1. Introduction

Primary liver cancer is a common clinical malignant tumor characterized by early metastasis, rapid progression, and high morbidity and mortality, among which hepatocellular carcinoma (HCC) accounts for more than 90% [1]. HCC is a tumor with a rich blood supply, and its growth and metabolism require continuous angiogenesis. Being a topical issue in tumor study, angiogenesis and changes in tissue blood flow can be reflected via CT perfusion imaging by quantitative measurement of tissue perfusion [2]. It is worth noting that the activation of the serum vascular endothelial growth factor (VEGF) and basic fibroblast growth factor (BFGF) can promote the formation of new blood vessels, leading to tumor recurrence and metastasis [3]. Nevertheless, the research on relevant parameters of CT perfusion imaging remains less than sufficient [4]. To fill the gap, this study explored the correlation between CT perfusion parameters of primary liver cancer and tumor angiogenesis, with an aim to provide a route to evaluate tumor angiogenesis in vivo.

## 2. Materials and Methods

### 2.1. Baseline Data

One hundred patients with primary liver cancer who were treated in our hospital from June 2019 to June 2021 were enrolled as the observation group, and 90 patients with benign liver lesions during in the same time frame were recruited as the control group.

Participants were assessed as eligible if confirmed with primary liver cancer by pathological diagnosis or European Association of Liver Diseases (EA-SL) criteria [5] and with complete medical data.

Whereas, patients with hepatitis and liver cirrhosis, myelodysplastic syndrome and other blood system diseases, allergies to CTPI contrast agent, or cardiopulmonary insufficiency were excluded from the study.

The study protocol has been reviewed and approved by the ethic committee of our hospital with the approval number of 201901023. The baseline feature in the two groups such as gender, age, and other general conditions were well balanced.

### 2.2. Scanning Method

#### 2.2.1. Preparation before Scanning

250 ml of 2% meglumine aqueous solution was orally administered 10 minutes before the examination to fill the gastrointestinal tract and breath-holding training was performed using abdominal girdle.

#### 2.2.2. Equipment and Scanning Methods and Parameters

The equipment applied was GE revolution ES spiral CT. The patient was instructed to perform thoracic breathing exercises, and the specific was as follows. CT plain scan followed by CTPI examination was performed, needle was retained through cubital vein puncture, and contrast agent iomeprol 60 mL (400 mg iodine/mL) was injected at a rate of 4.5 mL/s; then, rapid dynamic scan was performed during which patient held breath; there were 26 groups of dynamic volume scanning that was divided into 3 groups, with interval of 2 s between each group; there were 11 sets of images in the first group, 7 in the second group, and 8 in the third group, and then, CTPI images were collected. The images were analyzed using the software of the CT diagnostic system, the region of interest (ROI) was delineated in the dual-input maximum slope mode, the time density curve (TDC) was mapped, and the related parameters were measured, including hepatic arterial perfusion (HAP), hepatic portal perfusion (HPP), total liver perfusion (TLP), liver arterial perfusion index (hepatic arterial perfusion index, HAPI), and portal vein perfusion index (hepatic portal perfusion index, HPPI), and perfusion parameters were measured 3 times, and the average value was taken.

### 2.3. Serological Index Examination

3 ml of fasting cubital median venous blood was drawn from all patients and centrifuged at low temperature at a speed of 2000 r/min for 15 min. Serum was extracted and stored in a −70°C freezer for testing. Assays were performed in strict accordance with the instructions of the VEGF and BFGF kits.

### 2.4. Statistical Analysis

All data analyses were performed with SPSS 27.0. The enumeration data were expressed as rate (%) and processed via the chi-square test; Measurement data were expressed as mean ± standard deviation and verified via the *t*-test; repeated measures were analyzed by variance analysis; Pearson correlation analysis was used for relationship analysis. All were tested at a significance level of 0.05 (2-sided).

## 3. Results

### 3.1. Baseline Data

There were 60 males and 30 females in the control group; the average age was (68.5 ± 7.6) years; disease classification: 71 cases of simple liver cysts and 19 cases of other benign liver lesions. There were 59 males and 41 females in the observation group, and the average age was (68.3 ± 7.1) years; liver cancer stage: 18 patients with stage I, 30 patients with stage II, 27 patients with stage III, and 25 patients with stage IV. They were well balanced prior to the enrollment (*P* > 0.05), as given in Table 1.

### 3.2. Perfusion Parameters

Compared to the control group, significantly higher HAP and lower HPP and TLP were detected in the observation group. The perfusion volume indexes of patients with different stages of liver cancer in the observation group were statistically different (*P* < 0.05), as given in Tables 2 and 3.

### 3.3. Perfusion Index

Compared to the control group, the observation group witnessed significantly higher HAPI and lower HPPI. There were statistically significant differences in the perfusion index of patients with different stages of primary liver cancer in the observation group (*P* < 0.05), as given in Tables 4 and 5.

### 3.4. Serum VEGF and BFGF

The serum VEGF and BFGF levels in the observation group were significantly higher than those in the control group, and the serum VEGF and BFGF levels in patients with different stages of primary liver cancer in the observation group were statistically different (*P* < 0.05), as given in Tables 6 and 7.

### 3.5. Correlation Analysis between CT Perfusion Imaging-Related Parameters and Serum VEGF and BFGF in Patients with Primary Liver Cancer

Pearson correlation analysis showed that HAP and HAPI were positively correlated with VEGF and BFGF (*P* < 0.05), and HPP, TLP, and HPPI were negatively correlated with VEGF and BFGF (*P* < 0.05), as given in Table 8.

## 4. Discussion

The indicators associated with the occurrence and development of liver cancer remain the heated topic in current research studies [6] due to its significance in the early diagnosis of the disease, formulation of treatment measures, and evaluation of clinical efficacy [7]. With the development of imaging technology and the progress of liver cancer treatment, the diagnosis of liver cancer via the morphological localization and characterization cannot match a rhythm. Because functional change bears the brunt of tumor progression before the pathological anatomical changes of the tumor, the growth and metastasis of the tumor depends on ongoing angiogenesis [8]. These neovascularizations cause changes in blood volume, and perfusion volume and changes in capillary permeability underlie the enhancement [9].

VEGF is a growth factor that acts specifically on vascular endothelial cells and serves as the most direct and most important positive regulator to promote angiogenesis [10]. It strongly induces angiogenesis and is closely related to the growth, invasion, metastasis, staging, and prognosis of liver cancer [11]. Scholars have confirmed that VEGF is expressed in hepatocytes and liver cancer cells, and the expression intensity of VEGF is related to angiogenesis and cell proliferation [12]. BFGF, a polypeptide growth factor with a molecular weight of 15-16 kd and consisting of 146 amino acids [13], is located on human chromosome 4. It is a mitogen and an important angiogenic factor for cells of mesodermal and ectodermal origin [14]. It exerts physiological effects by binding to the cell surface specific receptor FGFR. It has been reported that BFGF is strongly associated with the occurrence and development of tumors [15]. When the body is under ischemia and hypoxia, large quantities of BFGF can be released to promote the formation of new blood vessels and maintain the needs of tumor growth [16]. Multiple studies revealed a strong correlation between that serum VEGF and BFGF and tumor growth and metastasis, and they promote lymphangiogenesis and metastasis [17]. In spite of marked results obtained in numerous studies with respect to disease stage, metastasis, degree of differentiation, and lesion size, the relationship of the above CT perfusion imaging parameters in HCC patients is still questioned [18].

According to our results, the CT perfusion imaging-related parameters and serum VEGF and BFGF in patients with primary liver cancer were significantly different from those in patients with benign liver lesions, and the CT perfusion parameters and serum VEGF and BFGF levels in patients with different stages of primary liver cancer were different, which was because blood of foci in primary liver cancer is mainly supplied by the hepatic artery with especially fast flow velocity, thereby increasing the pressure [19, 20]. Significantly, Pearson correlation analysis showed that CT perfusion parameters were correlated with serum VEGF and BFGF levels. As such, we consider that there is an intense correlation between the indicators and primary liver cancer, benefiting the diagnosis and treatment of primary liver cancer. We thus infer that the higher the expression of serum VEGF and BFGF-related indexes in patients with primary liver cancer, the more serious the abnormal formation of blood vessels and lymphatic vessels, the more abnormal blood perfusion, and the more visible changes in liver parenchyma blood flow [21, 22].

In conclusion, CT perfusion parameters and serum VEGF and BFGF levels in patients with primary liver cancer are abnormally expressed, and there is a strong correlation between the two, which might benefit clinical diagnosis and treatment.

## Figures and Tables

**Table 1:** Comparison of general data of the two patients.

Groups	*n*	Gender (*n*)		Age (year)
		Male	Female	
Control group	90	60	30	68.5 ± 7.6
Observation group	100	59	41	68.3 ± 7.1
*t*/*χ*^2^		1.190		0.182
*P*		0.275		0.856

**Table 2:** Comparison of perfusion volume indexes between the two groups (mL/(min·100 mL)).

Groups	*n*	HAP	HPP	TLP
Control group	90	23.41 ± 3.36	76.58 ± 6.17	102.98 ± 11.23
Observation group	100	38.83 ± 4.57	41.42 ± 5.75	73.15 ± 7.25
*t*		26.258	40.620	21.965
*P*		≤0.001	≤0.001	≤0.001

**Table 3:** Comparison of perfusion volume indexes in patients with different stages of primary liver cancer in the observation group (mL/(min·100 mL)).

Groups	*n*	HAP	HPP	TLP
I	18	31.62 ± 2.54	49.59 ± 2.10	84.05 ± 2.72
II	30	37.14 ± 1.53	44.10 ± 1.67	76.21 ± 1.99
III	27	40.72 ± 0.69	40.05 ± 1.18	70.84 ± 1.29
IV	25	43.98 ± 1.98	33.79 ± 2.62	64.10 ± 3.61
*F*		200.487	261.704	247.405
*P*		≤0.001	≤0.001	≤0.001

**Table 4:** Comparison of perfusion index between the control group and observation group (%).

Groups	*n*	HAPI	HPPI
Control group	90	23.14 ± 3.08	76.74 ± 6.24
Observation group	100	52.23 ± 5.21	46.18 ± 5.29
*t*		46.209	36.489
*P*		≤0.001	≤0.001

**Table 5:** Comparison of perfusion indices in patients with different stages of primary liver cancer in the observation group (%).

Groups	*n*	HAPI	HPPI
I	18	44.26 ± 1.52	50.04 ± 2.83
II	30	49.98 ± 1.74	48.39 ± 1.33
III	27	54.28 ± 0.91	44.58 ± 0.88
IV	25	58.47 ± 2.51	39.58 ± 2.50
*F*		253.814	216.284
*P*		≤0.001	≤0.001

**Table 6:** Comparison of serum VEGF and BFGF between the control group and observation group (pg/mL).

Groups	*n*	VEGF	BFGF
Control group	90	71.31 ± 10.69	4.45 ± 1.31
Observation group	100	120.70 ± 16.06	8.58 ± 1.27
*t*		24.675	22.081
*P*		≤0.001	≤0.001

**Table 7:** Comparison of serum VEGF and BFGF levels in patients with different stages of primary liver cancer in the observation group.

Groups	*n*	VEGF	BFGF
I	18	96.73 ± 8.15	6.88 ± 0.68
II	30	114.01 ± 4.01	7.84 ± 0.17
III	27	125.08 ± 2.26	9.02 ± 0.40
IV	25	141.23 ± 6.63	10.19 ± 0.52
*F*		261.369	228.069
*P*		≤0.001	≤0.001

**Table 8:** Correlation analysis of CT perfusion imaging-related parameters and serum VEGF and BFGF in patients with primary liver cancer.

CT perfusion index	VEGF		BFGF	
	*r*	*P*	*r*	*P*
HAP	0.986	≤0.001	0.969	≤0.001
HPP	−0.992	≤0.001	−0.976	≤0.001
TLP	−0.993	≤0.001	−0.978	≤0.001
HAPI	0.983	≤0.001	0.972	≤0.001
HPPI	−0.995	≤0.001	−0.984	≤0.001

## Data Availability

The datasets used to support this study are available from the corresponding author upon request.
